# Structural validity of the Chronic Pain Coping Inventory—Brazilian version

**DOI:** 10.1371/journal.pone.0246294

**Published:** 2021-02-08

**Authors:** Layz Alves Ferreira Souza, Lilian Varanda Pereira, Louise Amália de Moura, Leidy-Johanna Rueda Díaz, Diná de Almeida Lopes Monteiro da Cruz, José Aparecido Da Silva

**Affiliations:** 1 College of Nursing, Federal University of Goiás, Goiânia, Goiás, Brazil; 2 College of Nursing, Universidad Industrial de Santander, Bucaramanga, Santander, Colombia; 3 College of Nursing, University of São Paulo, São Paulo, São Paulo, Brazil; 4 Department of Psychology, Federal University of Juiz de Fora, Juiz de Fora, Minas Gerais, Brazil; Hong Kong Polytechnic University, HONG KONG

## Abstract

**Background:**

The Chronic Pain Coping Inventory (CPCI) has been widely used to measure coping with pain, however, the psychometric properties of the Brazilian CPCI are unknown.

**Aim:**

To verify the validity and reliability of the CPCI-Brazilian version.

**Materials and methods:**

A sample of 705 outpatients with chronic pain participated in the study. Cronbach’s alpha, corrected item-total correlations, and confirmatory factor analysis were performed, using the method of Diagonally Weighted Least Squares.

**Results:**

Construct validity was supported with a factor loading range of 0.36–0.90 (9 factors) corroborating original loads. The final model had adequate fit with items 42 and 54 excluded, D.F = 2174, TLI = 0.96; CFI = 0.96 and RMSEA = 0.051(p = 0.067). Eight of the nine CPCI scales showed satisfactory reliability (Cronbach’s alpha ranged from 0.70 to 0.92). The Relaxation scale obtained a low alpha value (0.53).

**Conclusion:**

The CPCI-Brazilian version, after exclusion of items 42 and 54, is valid to measure chronic pain coping in Brazilian adults.

## Introduction

Pain is a type of stressor, usually perceived as harmful and aversive, that impacts the individual’s daily life and provokes changes that require coping (adjustment or adaptation) [1, 2], which in this context is characterized as the efforts that people go through to manage pain [2, 3].

Pain coping has been shown to interfere with pain outcomes [4], such as intensity [5–7], in addition to psychological and physical functioning, such as outcomes quality of life [8], depression [6, 9, 10], anxiety [9, 11] and disability [9, 12].

For example, the coping strategies (CS) of Exercising/Stretching and Coping Self-Statements have had a significant negative correlation with the Numerical Rating Scale of Pain [6, 13], and non-adaptative CS like Guarding, Resting, and Asking for assistance have been positively correlated with pain intensity [13]. These and other correlations between different CS and pain outcomes have been reported in literature [14–17].

Because of the importance of the CS to pain outcomes, a current challenge is measurement of coping with chronic pain. However, health professionals and clinicians need reliable and valid tools to measure this construct.

One of the most widely used measures of pain coping is the Chronic Pain Coping Inventory (CPCI) [18], an instrument developed by the Multidisciplinary Pain Management Program of the University of Washington. The purpose of the tool was to fill the existing gaps in pain coping measurement and to focus the instrument on strategies frequently used in pain management programs, such as relaxation and exercises [19, 20]. The authors proposed the instrument based on a critical review of coping theory literature and studies of other tools such as the Vanderbilt Pain Management Inventory and the Coping Strategies Questionnaire [2, 19, 21].

The initial version of the CPCI, published in 1995, had 64 items to assess the use of cognitive and behavioral coping strategies [19], but in 2001 a review excluded the "Medication Used" scale and included the scale "Pacing" [22]. The instrument came to be constituted by 70 items and was copyrighted by the Psychological Assessment Resources (PAR) [20].

The CPCI is capable of evaluating two coping dimensions (Illness-focused CS and Wellness-focused CS) through 70 items in nine scales (Guarding, Resting, Asking for assistance, Relaxation, Persistence in task, Exercise/Stretching, Pacing, Coping self-statements, and Seeking social support) [20].

This measure has been validated for populations in the following countries: United States [13–15, 19, 23, 24], Canada (French language) and France [25, 26], Canada (English language) [22, 27], Sweden [28], Spain [16], China [7, 10, 29], North Korea [17], Portugal [5], Italy [6], Poland [30] and the Netherlands [31]. In Brazil there is a transcultural adapted version of the CPCI but its psychometric properties have not been researched [32].

The validation studies of the CPCI were conducted with adults and older people [13, 26–28], with chronic pain in several body sites (lumbar, lumbopelvic, people with fibromyalgia, generalized pain) [10, 17, 30, 31], with outpatient or hospitalized patients [5, 24, 29].

In the first validation study of CPCI, the reliability (alpha coefficient) ranged from 0.70 to 0.93 and the test-retest stability ranged from 0.66 to 0.90 [19]. Further studies showed general satisfactory reliability to the scales of CPCI (alpha > 0.70) [6, 13, 16, 28, 31], but some other studies pointed to alpha values less than 0.7 for the scales of Task Persistence (alpha range 0.50–0.69) [7, 17, 30], Relaxation (alpha range 0.51–0.68) [17, 26, 30] and Coping self-statements (alpha = 0.69) [7].

CPCI validation studies have investigated the psychometric properties of this tool by construct validity, mainly using construct correlations with pain intensity, pain interference, depression, anxiety, quality of life and disability [5, 6, 10, 13–16, 19, 22, 24, 25, 27, 29, 30]. Also, researchers studied the CPCI properties by structural validity through Principal Component Analysis [27], Exploratory Factor Analysis [17] and Confirmatory Factor Analysis (CFA) [6, 7, 16, 26] which presented the Root Mean Square Error of Approximation (RMSEA) values of the models ranging from 0.01 to 0.5 and the Comparative Adjustment Index (CFI) with values between 0.99 and 0.81, showing appropriate psychometric parameters [6, 7, 16, 26].

The use of the CPCI can improve clinical practice and studies around pain and help to explain some differences in the adjustment of people to the experience of pain [2, 33]. Moreover, chronic pain coping measurement can support pain management with non-adaptive CS that enhance emotional and physical health and improve psychological symptoms [3].

Given the relevance of measuring the pain coping construct, this study aimed to analyze the internal consistency and to perform a confirmatory factor analysis of the Brazilian version of the CPCI.

## Material and methods

### Design and setting

The CPCI has been adapted cross-culturally in Brazil [32], but without validation. For this, we proposed a methodological study to validate the Chronic Pain Coping Inventory (CPCI-Brazilian version). Methodological designs allow the development and validation of instruments and support new research methods [34, 35].

For the validation study of the instrument, we used the CFA, considering that the nine factors solution of the instrument are well established in the literature [19, 20, 22] and its results could show the adjustments of the set of items to the initially proposed theory [2, 36].

### Sample

A sample of 705 outpatients in neurology, orthopedics, physiatrics and rheumatology specialties of a university hospital in the Brazilian Midwest were recruited to the study, meeting the criterion of a minimum of 10 people per item for CFA [37, 38], considering the CPCI an instrument with 70 items. The research was conducted between November 2016 and December 2017 and the inclusion criteria for the sample were: chronic nonspecific pain (i.e., lasting continuously for ≥ 6 months) [39]; age > 18 years; and fluency in Brazilian Portuguese. The exclusion criteria were patients who could not verbalize or needed a proxy (for example, a caregiver) to answer the tool [40], those with a score ≤ 13 on the Mini-Mental State Examination (MMSE); and those who presented difficulties in the measurement tasks.

The cut-off point of ≤ 13 in MMSE was adopted considering a study that explored functional illiteracy in Brazil and showed that, after completing the final years of elementary school (approximately 8 years of study), 53% of people are in conditions similar to those who are illiterate [41]. Furthermore, another Brazilian study showed that the MMSE must have scores adjusted to the reality of the country, which means that in those who are illiterate, cognitive impairment can be considered when MMSE scores are ≤ 13 [42]. In the present study, education of the sample was expressed in years of study and ranged from 0 to 25 years, MD = 7.66 (±4.52).

Looking at the average level of education in the study sample exposes conditions of functional illiteracy, therefore an MMSE score was adopted, adjusted for people who are illiterate (cognitive impairment ≤ 13). Even so, 162 participants (22.97%) presented cognitive impairment but completed the measurement tasks without difficulties.

The study sample had a mean age of 53.81 (±14.26), MIN = 18 years and MAX = 89 years. They had, on average, a monthly family income of U$522.31 (±379.46). Descriptive statistics of the sample can be view in Table 1.

**Table 1:** Sociodemographic description and characterization of pain.

	n	%
**Age group**		
18–59 years	429	60.9
60 years or older	276	39.1
**Sex**		
Male	223	31.6
Female	482	68.4
**Marital status**		
With partner	378	53.8
Single	324	46.2
**Time living with pain**		
6 to 11 months	57	8.1
1 to 5 years	216	30.8
6 to 10 years	135	19.3
More than 10 years	293	41.8
**Main sites of pain**		
Head	141	20.0
Cervical	181	25.7
Upper limbs	398	56.5
Chest	208	29.5
Low back	386	54.8
Hip and pelvis	126	17.9
Lower members	544	77.2

### Procedures

Data were collected by seven trained interviewers, composed of nurses and one nutritionist. The training consisted of 20 hours of face-to-face meetings, coordinated by the main researcher. An instruction manual was given to each collector detailing the form of data collection for the entire instrument. Then, data collection training workshops were held among the interviewers. Finally, each collector performed eight hours of data collection supervised by the main researcher, who intervened and guided the conduct of the interviewers, when necessary. The data collected during training were not used in the present study.

After the outpatients registered their presence at the clinic, the interviewers approached them, checked if they met the inclusion criteria, invited them to participate in the study and if accepted, they were provided with a written informed consent form. The data was collected by a structured interview in the clinic waiting room, in an appropriate and private place. Psychological Assessment Resources (PAR), which owns the copyright to the CPCI, granted permission to use the CPCI-Brazilian version in this study, and it was approved by the Research Ethics Committee of the Federal University of Goiás under protocol 1.339.810. All patients provided written informed consent to participate, following the ethical precepts of the Declaration of Helsinki.

### Measures

The CPCI consists of 70 items that should be answered based on the number of days (zero to seven) a person used a particular CS in the past week. The sum of the items for each scale is the score for that type of CS. Higher values indicate higher levels of use of that CS type. The items of the CPCI are distributed according to two domains and nine scales.

The illness-Focused Coping domain includes the scales of Guarding (items 12, 16, 36, 38, 42, 44, 50, 52 and 60), Resting (items 5, 8, 20, 43, 51, 63 and 70) and Asking for Assistance (items 10, 27, 46 and 68). The Guarding scale refers to any restriction on the use or movement of any part of the body. Resting is the action of resting due to pain, such as lying down, sitting down, or going to a dark or silent place. And the Asking for assistance scale evaluate how often the person requests help with an activity when he/she are in pain, such as home chores or picking something up [20].

The domain of Wellness-Focused Coping is composed by the scales of Seeking social support (items 6, 9, 17, 22, 24, 48, 57 and 61), Coping self-statements (items 11, 15, 21, 23, 25, 29, 32, 40, 49, 53 and 58), Exercise/Stretching (items 3, 14, 19, 28, 31, 35, 41, 47, 56, 59, 65 and 66), Relaxation (items 1, 13, 26, 33, 39, 54 and 64), Task persistence (items 2, 4, 30, 37, 55 and 69) and Pacing (items 7, 18, 34, 45, 62 and 67) [20]. The Seeking social support dimension is characterized by actions such as talking or spending time with a friend or loved one when in pain (the focus of the conversation may or may not be the pain). Coping self-statements are purposeful positive thoughts that inspire hope. Exercise/Stretching scale is the commitment to some activity for muscle strengthening or stretching. Stretching activities should be continued for at least 10 seconds. In the case of exercises, the person must perform them to strengthen a specific muscle group or for aerobic conditioning purposes for at least 15 minutes. The Relaxation scale is the use of strategies such as meditation, listening to music, progressive muscle relaxation, diaphragmatic breathing, mental images, hypnosis, among others. Task Persistence is the tendency to maintain activities normally, despite the pain. And Pacing is the action of changing the rhythm of activities, such as performing them more slowly, taking breaks, or maintaining a different rhythm than usual [20].

The scores of the scales can be seen in Table 2.

**Table 2:** CPCI scales scores (0–7), Brazilian version.

CPCI Scales (n. items)	MD	SD
Relaxation (7)	1.64	1.28
Task Persistence (6)	4.27	1.90
Exercise/Stretching (12)	1.53	1.81
Seeking Social Support (8)	2.37	1.76
Pacing (6)	4.06	2.25
Coping Self-statements (11)	4.27	1.81
Guarding (9)	3.30	1.83
Asking for Assistance (4)	2.23	2.22
Resting (7)	3.21	1.82

CPCI, Chronic Pain Coping Inventory; CS, Coping strategies.

### Data analysis

Descriptive analyzes (frequencies, standard deviation, averages, and medians) were performed by IBM® SPSS Statistics® version 20.0, and the CFA was executed in software R (version 3.4.1). Less than 1% of the data were missing, therefore, an item mean was used to input missing values.

The reliability coefficient for each scale and domains were calculated using Cronbach’s alpha and corrected item-total correlations. Cronbach’s α values > 0.70 [43] and correlation values > 0.20 [44] were considered satisfactory.

The estimation method Diagonally Weighted Least Squares (DWLS) was performed, as the variables in the study did not present a normal distribution, since CPCI is a discrete and limited scale [45]. To verify the data fit to the CFA, the presence of outliers was analyzed (i.e., data tabulation errors or coding failures, observations arising from an extraordinary event, extraordinary observations for which the researcher does not have an explanation, and observations that are in the usual range of values for each variable but are unique in their combination of values between variables). The multivariate outliers were diagnosed based on the Mahalanobis D^2^ measurement [45].

After the analysis of outliers, the CFA continued, and items with factor loads less than 0.30 were eliminated from the final analysis because they undermined the reach of the basic assumptions for the validity and quality of the statistical model [38]. Fit to the CFA model was considered adequate with Comparative Adjustment Index (CFI) values greater than 0.80 [47, 48], Tucker-Lewis Index (TLI) greater than 0.80 [46, 47], and the Root Mean Square Error of Approximation (RMSEA) less than 0.10, with an ideal 0.05 value being expected [48].

## Results

### Reliability assessment

Psychometric properties according to the reliability of the instrument in each scale and by domains can be found in Table 3.

**Table 3:** CPCI reliability coefficients, Brazilian version.

CPCI Scales (n. items)	Cronbach’s alpha	Inter-item correlation mean
Relaxation (7)	.53	.13
Task Persistence (6)	.75	.33
Exercise/Stretching (12)	.92	.49
Seeking Social Support (8)	.81	.35
Pacing (6)	.84	.46
Coping Self-statements (11)	.86	.35
Guarding (9)	.76	.26
Asking for Assistance (4)	.81	.51
Resting (7)	.70	.25
**CPCI Domains**		
Wellness-focused CS (50)	.90	.14
Illness-focused CS (20)	.83	.19

CPCI, Chronic Pain Coping Inventory; CS, Coping strategies.

### Confirmatory factor analysis

Table 4 presents the cross-factor loads of the scales for the initial model. It is possible to observe that no item has a larger cross-factor load with another construct than with its original one. Therefore, all items were considered adequate for their respectivscales.

**Table 4:** Cross-factor loadings of the CPCI-Brazilian version.

Scale	Item	RE	TP	ES	SSS	PA	CSS	GU	AA	RES
Relaxation	1	**.45**	.08	.09	.10	.14	.27	.15	.01	.09
	13	**.65**	.04	.39	.10	.18	.27	.16	.05	.16
	26	**.43**	.19	.12	.14	.14	.25	.08	.11	.16
	33	**.36**	.02	.13	.13	.10	.09	.03	.03	.08
	39	**.53**	.05	.17	.11	.20	.27	.05	.08	.03
	54	**.28**	-.01	-.03	.10	-.02	.03	.04	.08	.11
	64	**.59**	.06	.26	.11	.19	.26	.24	.16	.14
Task Persistence	2	.07	**.73**	.05	-.01	.22	.20	-.07	-.03	-.11
	4	.14	**.59**	.12	.04	.21	.24	.02	.05	.00
	30	.06	**.74**	.08	-.08	.17	.17	-.17	-.14	-.17
	37	.09	**.50**	.05	.10	.20	.16	.00	.04	.08
	55	.25	**.85**	.15	.03	.32	.44	.13	.04	.00
	69	.06	**.83**	.06	-.03	.24	.24	-.11	-.12	-.14
Exercise/Stretching	3	.28	.09	**.83**	.01	.12	.09	-.01	.02	.00
	14	.30	.05	**.84**	.06	.12	.12	.03	.04	.06
	19	.35	.10	**.85**	.09	.18	.19	-.03	.09	.05
	28	.30	.07	**.87**	.10	.11	.10	-.01	.06	.06
	31	.37	.11	**.88**	.08	.15	.17	-.01	.05	.02
Exercise/Stretching	35	.21	.06	**.70**	.21	.05	.09	-.08	.01	.10
	41	.26	.01	**.80**	.11	.10	.12	.02	.02	.08
	47	.27	.06	**.85**	.11	.11	.11	-.07	.01	.07
	56	.21	.09	**.80**	.08	.10	.06	.01	.10	.09
	59	.25	.12	**.82**	.03	.14	.10	.00	-.02	.02
	65	.27	.09	**.88**	.08	.11	.13	-.01	.02	.04
	66	.29	.12	**.90**	.03	.10	.11	-.04	.02	.00
Seeking Social Support	6	.04	-.08	-.02	**.63**	.08	.04	.02	.09	.36
	9	.22	.07	.11	**.70**	.21	.26	.10	.19	.28
	17	.13	-.04	.04	**.76**	.20	.24	.23	.33	.31
	22	.09	.01	.09	**.73**	.19	.23	.08	.25	.31
	24	.18	.10	.08	**.70**	.18	.25	.08	.25	.25
	48	.13	-.05	.10	**.82**	.20	.22	.07	.24	.34
	57	.18	.02	.06	**.71**	.20	.19	.05	.20	.27
	61	.13	.00	.02	**.65**	.19	.22	.19	.23	.28
Pacing	7	.27	.17	.08	.24	**.67**	.26	.25	.17	.23
	18	.23	.30	.16	.24	**.84**	.33	.19	.18	.15
	34	.23	.11	.05	.25	**.69**	.25	.30	.20	.27
	45	.23	.31	.16	.17	**.90**	.32	.27	.19	.13
	62	.19	.23	.12	.19	**.89**	.29	.25	.18	.15
	67	.18	.25	.13	.19	**.77**	.29	.24	.14	.16
Coping Self-statements	11	.15	.17	.04	.20	.28	**.47**	.18	.18	.13
	15	.29	.20	.14	.22	.26	**.74**	.16	.05	.10
	21	.29	.16	.09	.19	.24	**.76**	.25	.07	.09
	23	.30	.26	.12	.22	.35	**.67**	.15	.06	.12
	25	.26	.25	.13	.20	.21	**.73**	.09	.01	.07
	29	.33	.20	.13	.18	.26	**.75**	.15	.08	.10
	32	.30	.18	.09	.26	.20	**.65**	.22	.15	.17
	40	.34	.27	.13	.18	.34	**.69**	.19	.06	.08
	49	.29	.22	.10	.11	.23	**.79**	.19	.02	.05
	53	.32	.20	.08	.29	.24	**.69**	.22	.12	.18
	58	.26	.20	.08	.21	.19	**.71**	.15	.13	.10
Guarding	12	.15	-.14	.02	.23	.15	.15	**.55**	.29	.20
	16	.21	.01	.05	.06	.24	.18	**.62**	.27	.15
	36	.16	-.04	-.09	.11	.28	.19	**.72**	.25	.31
	38	.13	-.04	-.07	.00	.14	.17	**.42**	.11	.08
	42	.22	-.01	.14	.05	.07	.13	**.32**	.14	.04
	44	.20	.06	.02	.06	.23	.22	**.66**	.18	.21
	50	.16	-.05	.00	.18	.26	.17	**.74**	.18	.46
	52	.14	-.05	.00	.08	.15	.19	**.72**	.33	.27
	60	.01	-.22	-.07	.14	.15	.07	**.64**	.30	.33
Asking for Assistance	10	.12	-.05	.01	.33	.16	.09	.25	**.83**	.27
	27	.09	-.07	.03	.27	.17	.08	.28	**.86**	.25
	46	.14	-.03	.07	.25	.25	.15	.35	**.77**	.20
	68	.11	-.06	.03	.26	.17	.09	.37	**.77**	.29
Resting	5	.15	-.10	.05	.32	.10	.08	.20	.16	**.66**
	8	.06	-.05	-.07	.28	.20	.10	.22	.21	**.55**
	20	.17	-.05	.08	.26	.14	.13	.30	.21	**.67**
	43	.14	-.02	.10	.26	.21	.13	.23	.19	**.51**
	51	.12	-.12	.06	.32	.17	.08	.34	.23	**.73**
	63	.19	-.14	.02	.26	.06	.12	.29	.20	**.58**
	70	.06	.04	-.05	.21	.17	.12	.16	.14	**.41**

RE, Relaxation; TP, Task persistence; ES, Exercise/stretching; SSS, Seeking social support; PA, Pacing; CSS, Coping self-statements; GU, Guarding; AA, Asking for assistance; RES, Resting.

In the analysis of outliers, no value was found outside the range of its respective variable. When analyzing the presence of univariate outliers, 87 (17.6%) observations were considered atypical. For multivariate outliers, no atypical individual was found. Considering that the observations of these outliers are valid cases of the population, it was decided not to exclude any of them.

The CFA proceeded using the DWLS method, pointing out the need to exclude item 54 (use of self-hypnosis) of the relaxation scale, because it has a factorial load less than 0.30, and item 42 (hold part of the body in a special position), because it contains in the confidence interval, a factorial load less than 0.30. In the final model, all otherscale items presented factorial loads > 0.30 (Table 5).

**Table 5:** Confirmatory factorial analysis of the CPCI scales, Brazilian version.

Scales		Initial Model		Final Model	
	Items	95%CI	F.L.	95%CI	F.L.
Relaxation	1	[.41; .49]	.45	[.41; .49]	.45
	13	[.61; .69]	.65	[.61; .69]	.65
	26	[.39; .47]	.43	[.39; .47]	.43
	33	[.32; .40]	.36	[.32; .40]	.36
	39	[.48; .57]	.53	[.48; .57]	.53
	54	[.21; .34]	.28	Excluded	-
	64	[.55; .63]	.59	[.54; .63]	.58
Task Persistence	2	[.69; .76]	.73	[.69; .76]	.73
	4	[.55; .64]	.59	[.55; .64]	.59
	30	[.71; .78]	.74	[.71; .78]	.74
	37	[.45; .54]	.50	[.45; .54]	.50
	55	[.81; .90]	.85	[.81; .90]	.86
	69	[.79; .87]	.83	[.79; .87]	.83
Pacing	7	[.64; .70]	.67	[.64; .70]	.67
	18	[.82; .87]	.84	[.82; .87]	.84
	34	[.66; .72]	.69	[.66; .72]	.69
	45	[.87; .92]	.90	[.87; .92]	.90
	62	[.87; .91]	.89	[.87; .91]	.89
	67	[.74; .79]	.77	[.74; .79]	.77
Exercise/Stretching	3	[.81; .85]	.83	[.81; .85]	.83
	14	[.82; .86]	.84	[.82; .86]	.84
	19	[.83; .87]	.85	[.83; .87]	.85
	28	[.85; .89]	.87	[.85; .89]	.87
	31	[.86; .90]	.88	[.86; .90]	.88
	35	[.67; .72]	.70	[.66; .72]	.69
	41	[.77; .82]	.80	[.77; .82]	.80
	47	[.83; .87]	.85	[.83; .87]	.85
	56	[.77; .83]	.80	[.77; .82]	.80
	59	[.80; .84]	.82	[.80; .84]	.82
	65	[.86; .90]	.88	[.86; .90]	.88
	66	[.88; .92]	.90	[.88; .92]	.90
Seeking social support	6	[.60; .67]	.63	[.60; .67]	.63
	9	[.67; .73]	.70	[.67; .73]	.70
	17	[.72; .79]	.76	[.72; .79]	.76
	22	[.70; .76]	.73	[.70; .76]	.73
Seeking social support	24	[.66; .74]	.70	[.66; .74]	.70
	48	[.79; .85]	.82	[.79; .85]	.82
	57	[.68; .74]	.71	[.68; .74]	.71
Coping Self-statements	11	[.44; .50]	.47	[.45; .50]	.48
	15	[.71; .77]	.74	[.71; .77]	.74
	21	[.74; .79]	.76	[.73; .79]	.76
	23	[.64; .70]	.67	[.64; .70]	.67
	25	[.70; .76]	.73	[.70; .76]	.73
	29	[.72; .78]	.75	[.72; .78]	.75
	32	[.62; .68]	.65	[.62; .68]	.65
	40	[.66; .72]	.69	[.66; .72]	.69
	49	[.76; .81]	.79	[.76; .81]	.79
	53	[.67; .72]	.69	[.67; .72]	.69
	58	[.68; .73]	.71	[.68; .73]	.71
Guarding	12	[.51; .59]	.55	[.49; .57]	.53
	16	[.58; .66]	.62	[.58; .65]	.61
	36	[.68; .75]	.72	[.69; .76]	.72
	38	[.39; .46]	.42	[.38; .45]	.42
	42	[.28; .35]	.32	Excluded	-
	44	[.63; .70]	.66	[.62; .70]	.66
	50	[.70; .77]	.74	[.70; .78]	.74
	52	[.68; .76]	.72	[.68; .76]	.72
	60	[.61; .67]	.64	[.61; .68]	.65
Resting	5	[.62; .69]	.66	[.62; .69]	.66
	8	[.52; .59]	.55	[.52; .59]	.56
	20	[.63; .71]	.67	[.63; .70]	.67
	43	[.47; .55]	.51	[.47; .55]	.51
	51	[.69; .77]	.73	[.69; .77]	.73
	63	[.54; .61]	.58	[.54; .61]	.57
	70	[.37; .45]	.41	[.37; .44]	.41
Asking for assistance	10	[.80; .86]	.83	[.80; .86]	.83
	27	[.82; .89]	.86	[.82; .89]	.86
	46	[.74; .81]	.77	[.74; .81]	.77
	68	[.74; .81]	.77	[.74; .81]	.77

95%CI, 95% Confidence interval; F.L., Factor loading

The path-map of structural equation modeling can be viewed in Figs 1–9.

**Fig 1:** Path map of Relaxation scale.

**Fig 2:** Path map of Task Persistence scale.

**Fig 3:** Path map of Exercise/Stretching scale.

**Fig 4:** Path map of Seeking social support scale.

**Fig 5:** Path map of Coping Self-statements scale.

**Fig 6:** Path map of Pacing scale.

**Fig 7:** Path map of Resting scale.

**Fig 8:** Path map of Guarding scale.

**Fig 9:** Path map of Asking for assistance scale.

In analysis of both models, it was verified that TLI and CFI values were higher than 0.95 (TLI = 0.96 and CFI = 0.96) and RMSEA value of 0.051 [0.050; 0.053], below the limit of 0.10, which indicates a good adjustment of the CFA model performed (Table 6).

**Table 6:** Adjustment parameters of the CPCI-Brazilian version to the CFA model.

Adjustment Quality Measures	Initial Model	Final Model
	DWLS	DWLS
D.F.	2309	2174
TLI	.96	.96
CFI	.96	.96
RMSEA	.052 [.050; .053]	.051[.050; .053]
p-value (RMSEA)	.025	.067

D.F., Degrees of Freedom; TLI, Tucker-Lewis Index; CFI, Comparative Fit Index; RMSEA, Root Mean Square Error of Approximation; DWLS, Diagonally Weighted Least Squares.

## Discussion

Analysis of the crossed factorial loads showed that no item had a larger factorial load in another construct than that of its origin, indicating the suitability of the items to their original constructs. An item saturation ≥ 0.3 explains approximately 10% of the explained variance of the factor analyzed, supporting the results obtained with the theory of the instrument [2, 14, 19].

In general, previous studies of the CPCI support the results of this study regarding the analysis of the factorial load factor matrix. The CFA of CPCI-64 items developed with American [14] and Canadian patients [27], as well as the CFA of CPCI-70 items Dutch version, among people with fibromyalgia [31], confirmed the saturation of CPCI items to their source. A minor exception occurred in the study in Canada, which identified some items with a larger factorial load in a scale other than the original one, which were: 24 (listening to music to relax), 48 (avoiding some physical activities), 39 (holding part of the body in a special position), 56 (avoid activities), 11 (avoid using part of the body) and 1 (imagine image to relax) [27].

During the CFA process of the CPCI-Brazilian version, two items were identified that did not reach a satisfactory factorial load (CF≥0.30, also considering their confidence interval): 54 (use self-hypnosis, CF = 0.28, CI = 0.21–0.34) and 42 (hold body part in special position, CF = 0.32, CI = 0.28–0.35). Nevertheless, the elimination of these items improved the results of the validity test.

Item 54 (use self-hypnosis) is worldwide known as an item with saturation problems, as occurred in Canadian [26], French [26] and Spanish [16] studies. Possibly, the lack of orientation, knowledge, and information about the practice of self-hypnosis among Brazilians may have contributed to the misfit of item 54. Hypnosis has been highlighted in the literature as an alternative for the non-pharmacological management of pain [49, 50], however, in clinical practice there is still skepticism on the part of professionals regarding the effectiveness of this therapy.

Item 42 (hold body part in special position), although saturated 0.32, obtained confidence interval < 0.3, and was excluded from the analysis. An exploratory study that used the Analysis of Principal Components in a Canadian sample pointed to a factorial load of 0.24 of this item in the guarding scale; on the other hand, it saturated 0.30 in resting and 0.37 in the asking for assistancescales [27]. This item was not identified with problems in its saturation in any of the CPCI validation studies that carried out confirmatory factor analysis [6, 14, 16, 31]. Although these findings partially corroborate this study, the revision or reformulation of both items is suggested for future research, since this is the first investigation in Brazil.

The low saturation in item 42 (hold part of the body in a special position) can be explained by the high frequency of reports of pain in the lower back (54.8%—Table 1) as well as the fact that the coping strategies of the "Task persistence" have been the most used (MD = 4.27), after all, immobilizing part of the body can hinder the performance of tasks.

The final CFA model of the CPCI-Brazilian version (with items 42 and 54 excluded) showed adequate adjustment with RMSEA(CI) = 0.051(0.050–0.053) and CFI = 0.96, confirming the structure in 9 scales, these being conceptually homogeneous. The validation parameters of the Brazilian validation were better than other studies, such as the validation of the Spanish version of the CPCI (42 items) in 402 people with fibromyalgia who found general adjustment of the CFA with RMSEA(CI) = 0.059 (0.057–0.061) and CFI = 0.81, being necessary the exclusion of item 33 (use self-hypnosis to relax) [16]. In the CFA of the CPCI (64 items) with 439 Canadians (French-speaking) and 388 French, partial adjustments were similar, RMSEA(CI) = 0.05(0.049–0.052) and CFI = 0.82 [26]. In the Dutch version of the CPCI-70 the final model adjustment presented RMSEA(CI) = 0.04 (0.03–0.04) and CFI = 0.88, and no item was excluded [31]. Perhaps this difference in parameters between the present study and the others mentioned may have occurred due to the size of the sample studied in the current study, which was bigger than the other studies. Furthermore, these studies were performed on different patient groups, which also could explain the differences in results.

This study also tested the internal consistency of the CPCI-Brazilian version and showed that Cronbach’s alpha and Inter-item correlation mean values of scales were satisfactory, indicating an adequate fit and internal consistency, with the exception of the Relaxation scale which was considered low. The Exercise/Stretching scale had the highest value (α = 0.92).

The low reliability of the relaxation scale (α = 0.53) can be explained by the low inter-item correlation of the scale (0.13). In addition, the activities considered relaxing can be different among people, for example, listening to music can be relaxing for some and not for others.

One limitation of this study concerns the data collection was performed by seven collectors, and inter-rater reliability was not investigated, although all were trained for the measurement tasks required by the study. Furthermore, despite patients with cognitive impairment must be considered when Patient Reported Outcome Measures (PROMs) are evaluated, the presence of 162 subjects with cognitive impairment have might influenced the results.

In addition, future studies should also investigate test-retest reliability, since the CPCI has great potential to be used in clinical practice to evaluate multidisciplinary therapy in chronic pain.

This study provides the first valid instrument for measuring the coping of chronic pain among Brazilians and confirms the original factorial structure of the instrument [20]. Also, the present study, as far as is known, is one of the validation studies of CPCI with the largest number of people in the sample, which gives greater robustness to the data presented.

## Conclusion

The CPCI-Brazilian version (with items 42 and 54 excluded) showed adequate validity and acceptable reliability as a Brazilian technology for measurement of chronic pain coping.

### Clinical implications

The results of this study may contribute to the assessment and treatment of chronic pain in Brazilian patients. The use of this measure in the clinical context is promising, as it will allow health professionals to evaluate the already used CS and propose interventions for those which are maladaptive. In addition, the use of CPCI-Brazilian version provides the necessary subsidies to evaluate the efficacy of therapies, especially those based on cognitive-behavioral theory, such as the training of coping skills [51–54]. It is also a tool that can be used by any trained health professional, that has been shown to be effective in evaluating the management of chronic pain from a biopsychosocial perspective [52, 55, 56]. In education, the CPCI can be used to teach the students to identify the CS for chronic pain. Investigators can use the CPCI for measure coping in descriptive, analytical or experimental studies, as well, to design interventions to help adults cope more effectively with pain.

## Supporting information

S1 Data (XLSX)

## References

[1] Van DammeS, CrombezG, EcclestonC. Coping with pain: A motivational perspective. Pain. 2008;139(1):1–4. 10.1016/j.pain.2008.07.022 18755548

[2] JensenMP, TurnerJA, RomanoJM, KarolyP. Coping with chronic pain: a critical review of the literature. Pain. 1991;47(3):249–83. 10.1016/0304-3959(91)90216-K 1784498

[3] LazarusRS. Coping Theory and Research: Past, Present, and Future. 1993;247:234–47. 10.1097/00006842-199305000-00002 8346332

[4] MeintsSM, EdwardsRR. Evaluating psychosocial contributions to chronic pain outcomes. Prog Neuro-Psychopharmacology Biol Psychiatry. 2018;87:168–82. 10.1016/j.pnpbp.2018.01.017 29408484PMC6067990

[5] Ferreira-ValenteMA, Pais RibeiroJL, JensenMP, AlmeidaR. Coping with Chronic Musculoskeletal Pain in Portugal and in the United States: A Cross-Cultural Study. Pain Med. 2011;12(10):1470–80. 10.1111/j.1526-4637.2011.01208.x 21834916

[6] MonticoneM, FerranteS, GiorgiI, GalandraC, RoccaB, FotiC. Development of the Italian version of the 42-item Chronic Pain Coping Inventory, CPCI-I: Cross-cultural adaptation, factor analysis, reliability and validity. Qual Life Res. 2013;22(6):1459–65. 10.1007/s11136-012-0271-y 23011492

[7] WongWS, JensenMP, MakKH, TamBKH, FieldingR. Preliminary psychometric properties of the Chinese version of the Chronic Pain Coping Inventory (ChCPCI) in a Hong Kong Chinese population. J pain. 2010;11(7):672–80. 10.1016/j.jpain.2009.10.008 20015705

[8] Yazdi-RavandiS, TaslimiZ, JamshidianN, SaberiH, ShamsJ, HaghparastA. Prediction of Quality of life by Self-Efficacy, Pain Intensity and Pain Duration in Patient with Pain Disorders. Basic Clin Neurosci [Internet]. 2013;4(2):117–24. ; PMCID: PMC420253625337337PMC4202536

[9] BairdA, SheffieldD. The Relationship between Pain Beliefs and Physical and Mental Health Outcome Measures in Chronic Low Back Pain: Direct and Indirect Effects. Healthc (Basel, Switzerland). 2016;4(3). 10.3390/healthcare4030058 27548244PMC5041059

[10] ChangHY, YangYL, JensenMP, LeeCN, LaiYH. The experience of and coping with lumbopelvic pain among pregnant women in Taiwan. Pain Med. 2011;12(6):846–53. 10.1111/j.1526-4637.2011.01151.x 21676156

[11] HigginsNC, BaileySJ, LaChapelleDL, HarmanK, HadjistavropoulosT. Coping Styles, Pain Expressiveness, and Implicit Theories of Chronic Pain. J Psychol. 2014;149(7):737–50. 10.1080/00223980.2014.977759 25396698

[12] AlschulerKN, MoltonIR, JensenMP, RiddleDL. Prognostic value of coping strategies in a community-based sample of persons with chronic symptomatic knee osteoarthritis. Pain. 2013;154(12):2775–81. 10.1016/j.pain.2013.08.012 23969326PMC4298486

[13] ErsekM, TurnerJA, KempCA. Use of the chronic pain coping inventory to assess older adults’ pain coping strategies. J Pain. 2006;7(11):833–42. 10.1016/j.jpain.2006.04.002 17074625

[14] TanG, NguyenQ, AndersonKO, JensenM, ThornbyJ. Further validation of the chronic pain coping inventory. J Pain. 2005;6(1):29–40. 10.1016/j.jpain.2004.09.006 15629416

[15] RomanoJM, JensenMP, TurnerJA. The chronic pain coping inventory-42: Reliability and validity. Pain. 2003;104(1–2):65–73. 10.1016/s0304-3959(02)00466-9 12855315

[16] Garcia-CampayoJ, PascualA, AldaM, Gonzalez RamirezMT. Coping with fibromialgia: Usefulness of the Chronic Pain Coping Inventory-42. Pain. 2007;132(SUPPL. 1):68–76. 10.1016/j.pain.2007.02.013 17400387

[17] KoY-M, ParkW-B, LimJ-Y. Cross-cultural adaptation and clinimetric property of Korean version of the Chronic Pain Coping Inventory-42 in patients with chronic low back pain. Spine (Phila Pa 1976). 2010;35(6):666–71. 10.1097/BRS.0b013e3181ba7a78 20139807

[18] KatoT. Frequently Used Coping Scales: A Meta-Analysis. Stress Health. 2015;31(4):315–23. 10.1002/smi.2557 24338955

[19] JensenMMP, Turner JAJA, Romano JMJM, Strom SSE. The chronic pain coping inventory: development and preliminary validation. Pain. 1995;60(2):203–16. 10.1016/0304-3959(94)00118-X 7784106

[20] JensenM, TurnerJ, RomanoJ, NielsonW. Chronic Pain Coping Inventory: Professional Manual. 1st ed Lutz: Psychological Assessment Resources Inc; 2008.

[21] JensenMP, KarolyP. Control beliefs, coping efforts, and adjustment to chronic pain. J Consult Clin Psychol. 1991;59(3):431–8. 10.1037//0022-006x.59.3.431 2071728

[22] NielsonWR, JensenMP, HillML. An activity pacing scale for the chronic pain coping inventory: Development in a sample of patients with fibromyalgia syndrome. Pain. 2001;89(2–3):111–5. 10.1016/s0304-3959(00)00351-1 11166466

[23] JensenMP, KeefeFJ, LefebvreJC, RomanoJM, TurnerJA. One- and two-item measures of pain beliefs and coping strategies. Pain. 2003;104(3):453–69. 10.1016/S0304-3959(03)00076-9 12927618

[24] TanG, NguyenQ, CardinSA, JensenMP. Validating the use of two-item measures of pain beliefs and coping strategies for a veteran population. J Pain. 2006;7(4):252–60. 10.1016/j.jpain.2005.11.007 16618469

[25] TruchonM, CôtéD. Predictive validity of the Chronic Pain Coping Inventory in subacute low back pain. Pain. 2005;116(3):205–12. 10.1016/j.pain.2005.04.003 15927382

[26] TruchonM, CôtéD, IrachabalS, CoteD, IrachabalS. The Chronic Pain Coping Inventory: confirmatory factor analysis of the French version. BMC Musculoskelet Disord. 2006;7:13 10.1186/1471-2474-7-13 16478541PMC1386669

[27] HadjistavropoulosHD, MacLeodFK, AsmundsonGJG. Validation of the Chronic Pain Coping Inventory. Pain [Internet]. 1999;80:471–81. 10.1016/S0304-3959(98)00224-3 10342409

[28] Ektor-AndersenJ, ØrbækP, IsacssonSO. Behaviour-focused pain coping: Consistency and convergence to work capability of the Swedish version of the chronic pain coping inventory. J Rehabil Med. 2002;34(1):33–9. 10.1080/165019702317242686 11900260

[29] ChengS, CheungC, NgV, LimH, LeungK, ChanA, et al Factor structure, psychometric properties, and correlates of revised Chinese version of Chronic Pain Coping Inventory among chronic pain patients in Hong Kong. internet J Pain, Symptom Control Palliat Care. 2014;10(1):1–7. 10.5580/IJPSP.22410

[30] MisterskaE, JankowskiR, GlowackiM. Psychometric properties of the Polish language version of the chronic pain coping inventory-42 for patients treated surgically due to herniated lumbar discs and spondylotic changes. Med Sci Monit. 2014;20:789–801. 10.12659/MSM.889728 24824781PMC4031224

[31] KarsdorpPA, VlaeyenJWS. Active avoidance but not activity pacing is associated with disability in fibromyalgia. PAIN. 2009;147(1):29–35. 10.1016/j.pain.2009.10.002 19716234

[32] SouzaLAF, de ALM daCruz D, PereiraLV. Cross-cultural adaptation of Chronic Pain Coping Inventory—Brazilian version. Brazilian J Pain. 2018;1(2): 103–10. 10.5935/2595-0118.20180020

[33] TurkDCD, FillingimRRB, OhrbachR, Patel KV. Assessment of Psychosocial and Functional Impact of Chronic Pain. J Pain. 2016;17(9):T21–49. 10.1016/j.jpain.2016.02.006 27586830

[34] ArafatA, ChowdhuryH, QusarM, HafezM. Cross-cultural adaptation and psychometric validation of research instruments: A methodological review. J Behav Heal. 2016;5(3):129–36. 10.5455/jbh.20160615121755

[35] PolitDF, BeckC. Essentials of Nursing Research: Appraising Evidence for Nursing Practice 9th ed Philadelphia, USA: Wolters Kluwer; 2019 512 p.

[36] MuellerRO, HancockGR. Factor Analysis and Latent Structure, Confirmatory In: SmelserNJ, Baltes PBBT-IE of the S& BS, editors. Oxford: Pergamon; 2001;5239–44. 10.1016/B0-08-043076-7/00426-5

[37] ForeroC, Maydeu-OlivaresA, Gallardo-PujolD. Factor analysis with ordinal indicators: A monte carlo study comparing DWLS and ULS estimation. Struct Equ Model. 2009;16:625–41. 10.1080/10705510903203573.

[38] MvududuNH, SinkCA. Factor Analysis in Counseling Research and Practice. Couns Outcome Res Eval. 2013;4(2):75–98. 10.1177/2150137813494766

[39] MerskeyH, BogdukN. Classification of chronic pain In: Classification of Chronic Pain. second. Seattle: IASP Press; 1994 p. 1 10.1016/0304-3959(94)90180-5

[40] PetersenRC, CaraccioloB, BrayneC, GauthierS, JelicV, FratiglioniL. Mild cognitive impairment: a concept in evolution. J Intern Med. 2014;275(3):214–28. 10.1111/joim.12190 24605806PMC3967548

[41] Instituto Paulo Montenegro. Functional illiteracy indicator—INAF: Special study on literacy and the world of work. São Paulo; 2016.

[42] BertolucciPHF, BruckiSMD, CampacciSR, JulianoY. The Mini-Mental State Examination in an outpatient population: influence of literacy. Arq. Neuro-Psiquiatr.1994;52(1):1–7.doi: 10.1590/S0004282X19940001000018002795

[43] BlandJM, AltmanDG. Statistics Notes: Cronbach’s Alpha. BMJ Br Med J. 1997;314(7080):572 10.1136/bmj.314.7080.5729055718PMC2126061

[44] KlineP. A Handbook of Test Construction: Introduction to Psychometric Design. 1st ed New York: Routledge; 1986. 274 p.

[45] HairJ, BlackW, BabinB, AndersonR, TathamR. Multivariate Data Analysis. 8th ed Cengage; 2018.

[46] BentlerP. Comparative fit indexes in structural models. Psychol Bull. 1990;107(2). 10.1037/0033-2909.107.2.2382320703

[47] BentlerP, BonettD. Significance tests and goodness of fit in the analysis of covariance structures. Psychol Bull. 1980;88(3):588 10.1037/0033-2909.88.3.588

[48] SteigerJ, ShapiroA, BrowneM. On the multivariate asymptotic distribution of sequential chi-square statistics. Psychometrika. 1985;50(3):253–63. 10.1007/BF02294104

[49] JafarizadehH, LotfiM, AjoudaniF, KianiA, AlinejadV. Hypnosis for reduction of background pain and pain anxiety in men with burns: A blinded, randomised, placebo-controlled study. Burns. 2018;44(1):108–17. 10.1016/j.burns.2017.06.001 28801149

[50] ThompsonT, TerhuneDB, OramC, SharangparniJ, RoufR, SolmiM, et al The effectiveness of hypnosis for pain relief: A systematic review and meta-analysis of 85 controlled experimental trials. Neurosci Biobehav Rev. 2019;99:298–310. 10.1016/j.neubiorev.2019.02.013 30790634

[51] BroderickJE, KeefeFJ, BruckenthalP, JunghaenelDU, SchneiderS, SchwartzJE, et al Nurse practitioners can effectively deliver pain coping skills training to osteoarthritis patients with chronic pain: A randomized, controlled trial. Pain. 2014;155(9):1743–54. 10.1016/j.pain.2014.05.024 24865795PMC4171086

[52] RichardsonC, PooleH. Chronic pain and coping: a proposed role for nurses and nursing models. J Adv Nurs. 2001;34(5):659–67. 10.1046/j.1365-2648.2001.01795.x 11380734

[53] RiddleDL, KeefeFJ, NayWT, McKeeD, AttarianDE, JensenMP. Pain coping skills training for patients with elevated pain catastrophizing who are scheduled for knee arthroplasty: A quasi-experimental study. Arch Phys Med Rehabil. 2011;92(6):859–65. 10.1016/j.apmr.2011.01.003 21530943PMC3104058

[54] SchrubbeLA, RavytsSG, BenasBC, CampbellLC, CenéCW, CoffmanCJ, et al Pain coping skills training for African Americans with osteoarthritis (STAART): study protocol of a randomized controlled trial. BMC Musculoskelet Disord. 2016;17(1):359 10.1186/s12891-016-1217-2 27553385PMC4994196

[55] IsmailA, MooreC, AlshishaniN, YaseenK, AlshehriMA. Cognitive behavioural therapy and pain coping skills training for osteoarthritis knee pain management: a systematic review. J Phys Ther Sci. 2017;29(12):2228–35. 10.1589/jpts.29.2228 29643612PMC5890238

[56] NicholasM. Expanding Patients’ Access to Help in Managing Their Chronic Pain. Pain Clin Updat. 2015;23(1):1–8.

